This article has been retracted.

# Long Intergenic Nonprotein Coding RNA 00174 Aggravates Lung Squamous Cell Carcinoma Progression via MicroRNA-185-5p/Nuclear Factor IX axis

**DOI:** 10.1155/2022/9490827

**Published:** 2022-08-25

**Authors:** Peipei Gu, Lin Lin

**Affiliations:** Department of Thoracic Surgery, The No. 4 Hospital, No. 50 Shifan Road, Tianqiao District, Jinan, 250000 Shandong, China

## Abstract

Extensive studies have presented that long noncoding RNAs (lncRNAs) are closely implicated in the pathogenesis of various human malignancies, including lung squamous cell carcinoma (LUSC). This study explored the biological role and the underlying mechanism of long intergenic nonprotein coding RNA 00174 (LINC00174) in LUSC. LINC00174 expression was measured by reverse transcription quantitative real-time polymerase chain reaction (RT-qPCR). Both in vitro and in vivo experiments were conducted to determine LINC00174 function in LUSC. Mechanical assays were performed to investigate the molecular mechanism involving LINC00174 and related genes. LINC00174 expression was high in LUSC cells. Silencing of LINC00174 could restrain LUSC cells proliferation, migration, and invasion while promoting cell apoptosis. Mechanically, LINC00174 could interact with miR-185-5p to upregulate nuclear factor IX (NFIX), which was the direct target gene of miR-185-5p. Notably, NFIX elevation could rescue the repressing effect of LINC00174 silence on LUSC cell malignant behaviors. Our data suggested that LINC00174 aggravated LUSC progression via serving as a competing endogenous RNA (ceRNA) to sponge miR-185-5p and ultimately upregulate NFIX, which offered a promising novel target for LUSC therapy.

## 1. Introduction

Lung cancer is the most common malignant tumor, which occupies approximately 11.6% of all cancer cases. With high incidence and mortality rates, it is the leading cause of cancer-related mortality, accounting for about 18.4% of the total death cases [1]. Lung cancer is divided into two principle categories, namely, small cell lung cancer and non-small-cell lung cancer (NSCLC) [2]. Lung adenocarcinoma (LUAD) and lung squamous cell carcinoma (LUSC) are the two prevalent histological forms of NSCLC. LUSC is characterized by unfavorable clinical response, high relapse circumstances, and poor prognosis [3]. Hence, it is crucial to find novel genes implicated in the progression of LUSC, which may be targeted in clinical treatment.

As a group of noncoding RNAs longer than 200 nucleotides, long noncoding RNAs (lncRNAs) have been extensively studied for their important regulatory role in various cancers, because they could mediate gene expression at both transcriptional and posttranscriptional level [4]. Substantial research revealed that lncRNAs could play an essential role in pathologic processes. The dysregulated lncRNAs in cancers could exert profound effects on cellular activities, such as proliferation, apoptosis, and migration [5, 6]. Notably, the competing endogenous RNA (ceRNA) network has been extensively studied in the tumorigenesis processes. Increasing lncRNAs have been revealed to engage in ceRNA network at posttranscriptional level via acting as miRNA sponge. lncRNAs could competitively bind to shard miRNAs against mRNA and relive mRNA repressed by miRNA, thus increasing the corresponding protein levels [7]. Accumulating studies have uncovered a wide array of lncRNAs that are involved in the development and progression of LUSC [8]. Also, previous reports highlighted the clinical significance of targeting lncRNAs to affect the progression of LUSC [9, 10].

LINC00174 has been identified as an oncogene in colorectal carcinoma via regulating miR-1910-3p/TAZ axis [11]. However, its molecular role and underlying mechanism in LUSC still remain obscure. In present study, we aimed to determine the role of LINC00174 in LUSC progression. We also explored whether LINC00174 exerted its molecular function via ceRNA mechanism.

## 2. Materials and Methods

### 2.1. Cell Culture and Transfection

LUSC cells (SK-MES-1, NCI-H226, SW900, and NCI-H520) and normal pulmonary epithelial cell (BEAS-2B) were both procured from American Type Culture Collection (Rockville, Maryland). SK-MES-1 cells were cultivated in Eagle's minimum essential medium (EMEM). NCI-H226 and NCI-H520 cells were cultivated in RPMI-1640 medium. SW900 cells were cultivated in Leibovitz's L-15 medium. BEAS-2B cells were cultivated in BEGM (Lonza/Clonetics Corporation). All cell were cultured under the condition of 5% CO_2_ and 37°C. 10% fetal bovine serum (FBS; Gibco, Grand Island, NY) and 1% penicillin-streptomycin solution (Invitrogen) served as the medium supplements.

Cell transfection was implemented with Lipofectamine 3000 (Invitrogen) for 48 h. The two short hairpin RNAs (shRNAs) of LINC00174 and negative control (NC) sh-NC, the pcDNA3.1/nuclear factor IX (NFIX) and pcDNA3.1 as NC, the miR-185-5p mimics/inhibitor, and the NC mimics/inhibitor were procured from RiboBio (Guangzhou, China).

### 2.2. RNA Isolation and Reverse Transcription Quantitative Real-Time Polymerase Chain Reaction (RT-qPCR) [12]

Total RNA was isolated from LUSC cells in line with the standard method of TRIzol reagent (Invitrogen) and then converted into complementary DNA (cDNA). SYBR Green PCR Master Mix (Takara, Kyoto, Japan) was applied for qPCR experiment. Each gene expression level was calculated with quantitative 2^−*ΔΔ*CT^ method, with GAPDH and U6 as the standardized genes.

### 2.3. Colony Formation

LUSC cells were reaped after transfection and planted at a density of 500 cells/well in the 6-well plates. After fixation in 4% paraformaldehyde, colonies were treated with 0.1% crystal violet for determining the colony formation rate.

### 2.4. 5-Ethynyl-2′-Deoxyuridine (EdU) Assay

EdU assay was implemented as per the instruction of EdU incorporation assay kit (Ribobio) after cells were transfected with indicated plasmids. 100 *μ*L of 50 *μ*M EdU was added into the 96-well plates for 3 h of cell culture, followed by fixation and permeabilization. Nuclear staining of LUSC cells was performed with DAPI solution.

### 2.5. Terminal-Deoxynucleotidyl Transferase Mediated Nick End Labeling (TUNEL) Assay

Apoptotic LUSC cells were quantified by TUNEL assay using One-Step TUNEL Apoptosis Assay Kit (Beyotime, Shanghai, China) following the user's manual. DAPI was used to stain nuclei. The TUNEL-positive cells were determined after observation. The TUNEL-positive cell rate was analyzed with ImageJ.

### 2.6. Transwell Assays

Cell migration assay was achieved by use of the 24-well plate Transwell chamber with 8 *μ*m pores (Corning Company, New York). 50 *μ*L of Matrigel (Sigma-Aldrich Chemical Company, St Louis, MO) was put in the chamber for cell invasion assay. 4 × 10^4^ cells of SK-MES-1 or NCI-H520 in the serum-free medium were seeded into the upper chamber, while 650 *μ*L of complete medium was added to the lower chamber. Successfully migrated or invaded cells were then fixed in methanol and stained with 0.1% crystal violet. Images were collected under the inverted optical microscope. The number of cells was analyzed via ImageJ.

### 2.7. Subcellular Fractionation

1 × 10^6^ LUSC cells were initially prepared for isolating the cell nucleus and cell cytoplasm as per the user manual of PARIS™ Kit (Invitrogen). After washing and centrifuging, the levels of isolated RNAs (LINC00174, U6, and GAPDH) were assessed by RT-qPCR.

### 2.8. Fluorescence In Situ Hybridization (FISH)

The fixed LUSC cells in 4% formaldehyde were reaped after washing for incubating in hybridization buffer with the LINC00174 FISH probe (RiboBio) following the user guide. After being stained with Hoechst solution, the cells were observed through a FV1000 confocal laser microscope (Olympus, Tokyo, Japan). The probe sequence was listed in the Supplementary file.

### 2.9. Dual-Luciferase Reporter Assay

The wild-type (WT) and mutated (MUT) fragments of LINC00174 or NFIX 3′UTR covering the miR-150-5p binding sites were severally inserted to the downstream of Dual-Luciferase miRNA Target Expression Vector pmirGLO (Promega Corporation, Fitchburg, WI). Recombinant luciferase reporter vectors LINC00174 WT/MUT and AZIN1 3′UTR WT/MUT were cotransfected with miR-185-5p mimics or NC mimics into SK-MES-1 or NCI-H520 cells and then analyzed after 48 h by Dual-Luciferase Reporter Assay System (Promega).

### 2.10. RNA Pull Down

The sequences of LINC00174 were synthesized and biotin-labeled to construct Bio-LINC00174, followed by treatment with LUSC cell lysate acquired through RIPA buffer for 1 h. 50 *μ*l of streptavidin beads was then added, and the precipitations were collected by centrifugation, and RT-qPCR was followed.

### 2.11. RNA Binding Protein Immunoprecipitation (RIP) Analysis

The lysates of 1 × 10^7^ LUSC cells were acquired from RIP lysis buffer for immunoprecipitation with the antibody against human Ago2 or normal control IgG (Millipore, Bedford, MA) for 1 h. After incubation with beads, the purified RNAs were subjected to RT-qPCR analysis.

### 2.12. Western Blot

Total protein samples from LUSC cells were obtained for electrophoresis with 10% sodium dodecyl sulfate-polyacrylamide gel electrophoresis and then transferred onto polyvinylidene fluoride membranes. 5% nonfat milk was used to seal membranes. Primary antibodies against NFIX and GAPDH as control, as well as the appropriate secondary antibodies, were both purchased from Abcam (Cambridge, MA). Samples on the membranes were analyzed by enhanced chemiluminescence reagent (Santa Cruz Biotechnology, Santa Cruz, CA).

### 2.13. In Vivo Experiment

Male nude mice at 6 weeks old were procured from the National Laboratory Animal Center (Beijing, China) and maintained in the animal lab under specific pathogen free (SPF) grade, with the approval from the Animal Research Ethics Committee of the No. 4 Hospital. In vivo experiment was performed via subcutaneous injection of 5 × 10^6^ SK-MES-1 cells into nude mice (3 mice per group). Tumor volume was calculated every 4 days. 28 days after inoculation, tumors were carefully excised and weighed after mice were killed.

### 2.14. Statistical Analyses

Results were given as mean ± standard deviation of 3 or more biological independent assays. PRISM 6 (GraphPad, San Diego, CA) was applied to determine the statistical significance via one-way or two-way analysis of variance (ANOVA) and *t* test, with *P* value less than 0.05 as threshold.

## 3. Results

### 3.1. LINC00174 Depletion Suppresses Proliferation and Migration in LUSC Cells

We firstly used TCGA database to predict the correlation between LINC00174 and the overall survival of LUSC patients. We found that patients with high expression of LINC00174 were accompanied with short survival time. Then, we observed a significant higher expression of LINC00174 in LUSC cells (SK-MES-1, NCI-H226, SW900, and NCI-H520) compared with normal pulmonary epithelial cell (BEAS-2B) (Figure 1(a)). Afterwards, we knocked down LINC00174 in SK-MES-1 and NCI-H520 cells by transfecting two shRNAs against LINC00174 and applied RT-qPCR to verify the knockdown efficiency (Figure 1(b)). Subsequently, colony formation assay was performed, and the results indicated that LINC00174 silence could restrain the proliferation of SK-MES-1 and NCI-H520 cells (Figure 1(c)). It was further proved by EdU assay, as illustrated in Figure 1(d), EdU-positive cells decreased in response to LINC00174 depletion. In addition, we found that TUNEL-positive cell's rate increased with LINC00174 downregulation, indicating cell apoptosis was strengthened when LINC00174 was knocked down (Figure 1(e)). Moreover, knockdown of LINC00174 markedly impaired cell migration and invasion (Figures 1(f) and 1(g)). Therefore, it could be concluded that LINC00174 exacerbated LUSC cell proliferation, migration, and invasion but impeded LUSC cell apoptosis.

### 3.2. LINC00174 Binds to miR-185-5p in LUSC Cells

To probe into the regulatory mechanism, we continued to detect the subcellular location of LINC00174 in LUSC cells. As a result, LINC00174 was primarily situated in the cytoplasm (Figures 2(a) and 2(b)). As widely reported, cytoplasmic lncRNAs could bind to miRNAs and serve as miRNA sponge [13]. Hence, we searched on starBase (http://starbase.sysu.edu.cn) and found 5 potential miRNAs bound to LINC00174 under the screening condition of pan − cancer ≥ 10 (Figure 2(c)). Subsequently, we performed RNA pull down assay and found a significant combination between miR-185-5p and biotinylated LINC01174 (Figure 2(d)). We examined miR-185-5p expression and found that miR-185-5p expression was aberrantly lower in LUSC cells in comparison with BEAS-2B cells (Figure 2(e)). The putative binding sequences of miR-185-5p and LINC00174 and the corresponding mutant sequence of LINC00174 are shown in Figure 2(f). Furthermore, we overexpressed miR-185-5p in LUSC cells and found that miR-185-5p mimics could weaken the luciferase activity of LINC00174-WT while having no significant change on that of LINC00174-MUT (Figure 2(g)). Hence, it could be confirmed that LINC00174 bound to miR-185-5p in LUSC cells.

### 3.3. NFIX Is the Target Gene of miR-185-5p

miRNAs are widely reported to affect carcinogenesis by targeting specific downstream genes. Therefore, we continued to ravel out the target genes of miR-185-5p. By utilizing RNA22, micro T, and Target Scan tools, we found 8 potential targets of miR-185-5p (Figure 3(a)). We noticed that only the expression level of NFIX was reduced in SK-MES-1 and NCI-H520 cells after the transfection of miR-185-5pmimics (Figure 3(b)). Besides, NFIX was detected to be obviously overexpressed in LUSC cells (Figure 3(c)). Subsequently, RIP assay was performed, and the result manifested that enrichment of LINC00174, miR-185-5p, and NFIX were all substantial in Ago2 group compared with IgG group (Figure 3(d)). In addition, we found that putative binding sites between miR-185-5p and NFIX 3′UTR with mutant binding site were also designed (Figure 3(e)). Luciferase reporter assays showed that the luciferase activity of NFIX 3′UTR-WT was decreased significantly after miR-185-5p depletion (Figure 3(f)). More importantly, we found that the expression of NFIX was decreased after transfection ofsh-LINC00174 but was increased again when miR-150-5p inhibitor was cotransfected (Figure 3(g)). Therefore, LINC00174 positively modulated NFIX via binding to miR-150-5p.

### 3.4. LINC00174 Aggravates Lung Squamous Cell Carcinoma Progression via Upregulating NFIX

Finally, we performed rescue functional assays to verify whether LINC00174 facilitated LUSC progression via modulating NFIX. Preparedly, we increased the expression of NFIX inSK-MES-1 and NCI-H520 cells, and RT-qPCR proved that the overexpression efficiency was high enough (Figure 4(a)). Furthermore, we noticed that the reduced expression of NFIX caused by LINC00174 knockdown was elevated again after cotransfection of pcDNA3.1/NFIX (Figure 4(b)). Western blot also proved this result (Figure 4(c)). In colony formation and EdU assays, we observed that the repressing effect of sh-LINC00174#2 on cell proliferation was abolished by synchronous NFIX overexpression (Figures 4(d) and 4(e)). Besides, the facilitated cell apoptosis induced by sh-LINC00174#2 was counteracted by NFIX overexpression (Figure 4(f)). Moreover NFIX overexpression also recovered the inhibited migration and invasion resulted from LINC00174 depletion (Figures 4(g) and 4(h)). We also conducted in vivo experiments to further validate the function of LINC00174/NFIX axis in LUSC. Nude mice experiment results suggested that the tumor growth was much slower in sh-LINC00174#2-transfected group, but it was accelerated by upregulated NFIX (Figure 4(i)). The tumor volume and weight were measured to be lessened in the sh-LINC00174#2 group but were increased again after overexpressing NFIX (Figures 4(j) and 4(k)).

## 4. Discussion

It has been well documented that lncRNAs are critical regulators in human cancers, such as ovarian cancer, breast cancer, and prostate cancer [14–16]. The correlation between lncRNA and LUSC has been revealed [17]. Here, we initially found that LINC00174 was aberrantly high expressed in LUSC cells. Knockdown of LINC00174 could repress LUSC cell proliferation, migration, and invasion while facilitating LUSC apoptosis, indicating the carcinogenic role of LINC00174 in LUSC. It was inconsistent with the previous finding that LINC00174 promotes glioma progression via miR-152-3p/SLC2A1 axis [18] and that LINC00174 plays an oncogenic role in hepatocellular carcinoma [19].

To date, numerous lncRNAs have been found to act as miRNA sponges to affect downstream gene expression, thus influencing cancer progression. As reported previously, LINC00174 promotes chemoresistance of glioma cells via miR-138-5p/SOX9 axis [20]. LINC00174 sponges miR-1910-3p to increase colorectal carcinoma progression via influencing TAZ [11]. Consistently, our study found that LINC00174 was bound to miR-185-5p in LUSC cells. miR-185-5p functions as a tumor suppressor in many kinds of cancers, such as hepatocellular carcinoma [21] and glioma [22]. In addition, we found that miR-185-5p expression was low in LUSC cells.

Existing researches have verified that NFIX acts as an oncogene in many cancers, including pancreatic cancer [23] and gastric cancer [24]. Besides, a variety of miRNAs have been documented to affect cancer progression via targeting NFIX [25]. Herein, our study found that miR-185-5p directly targeted NFIX in LUSC cells. NFIX was positively regulated by LINC00174 and negatively regulated by miR-185-5p. It was validated that LINC00174 upregulated NFIX in LUSC cells via sponging miR-185-5p. In addition, in vitro and in vivo rescue experiments further confirmed that LINC00174 promoted LUSC cell growth and tumor growth via elevating NFIX expression. In summary, we firstly found that LINC00174 promoted LUSC cell proliferation and migration by regulating miR-185-5p/NFIX axis. Still, further research involving clinical samples should be conducted for confirming the clinical value of LINC00174 as a therapeutic target in LUSC. However, a more comprehensive understanding of LUSC at molecular level could be obtained from this study.

## Figures and Tables

**Figure 1:** LINC00174 depletion suppresses the malignant behaviors of LUSC cells. (a) RT-qPCR determined LINC00174 expression in LUSC cells and BEAS-2B. (b) The inhibitory efficiency of sh-LINC00174#1/2 was detected by RT-qPCR analysis. (c and d) Colony formation and EdU assays evaluated cell proliferation after knockdown of LINC00174. (e) TUNEL assay assessed LUSC cells apoptosis after silencing LINC00174. (f and g) Transwell migration and invasion assays were investigated cell migration and invasion ability after silencing LINC00174. ^∗∗^*P* < 0.01.

**Figure 2:** LINC00174 binds to miR-185-5p. (a and b) Subcellular fractionation and FISH assays were utilized to determine the cellular situation of LINC00174. (c) Possible miRNAs combined with LINC00174 were predicted from starBase. (d) RNA pull down assay was performed to study the affinity between LINC00174 and potential combinable miRNAs. (e) RT-qPCR analysis was performed to detect miR-185-5p expression in LUSC cells. (f) Binding sites between LINC00174 and miR-185-5p were displayed. (g) Luciferase reporter assays were performed to verify the interaction between LINC00174 and miR-185-5p. ^∗∗^*P* < 0.01.

**Figure 3:** NFIX is the target gene of miR-185-5p. (a) RNA22, micro T, and Target Scan tools predicted 8 potential targets of miR-185-5p. (b) RT-qPCR detected the expression of mRNA candidates after overexpressing miR-185-5p. (c) RT-qPCR evaluated NFIX expression in LUSC cells. (d) RIP assay detected the enrichment of LINC00174, miR-185-5p, and NFIX in anti-IgG and anti-Ago 2 groups. (e) Binding sites between miR-185-5p and NFIX 3′UTR were displayed. (f) Dual luciferase reporter assays determined the relationship between miR-185-5p and NFIX 3′UTR. (g) RT-qPCR analysis was performed to study the effects of sh-NC, sh-LINC00174#2, and sh-LINC00174#2+miR-185-5p inhibitor on NFIX expression. ^∗∗^*P* < 0.01.

**Figure 4:** LINC00174 aggravates LUSC progression via regulating NFIX. (a) RT-qPCR examined NFIX expression in LUSC cells after transfecting with pc DNA3.1 and pcDNA3.1/NFIX. Rescue assays were performed with LUSC cells after transfection of sh-NC, sh-LINC00174#2, and sh-LINC00174#2+pcDNA3.1/NFIX, respectively. (b and c) RT-qPCR and western blot determined the expression of NFIX. (d and e) Colony formation and EdU experiments detected the cell proliferation. (f) TUNEL assay detected the apoptosis. (g and h) Transwell assays detected the cell migration and invasion. (i) Xenograft tumor growth curve was shown. (j and k) Xenograft tumor volume and weight were measured. ^∗∗^*P* < 0.01.

## Data Availability

All data, models, and code generated or used during the study appear in the submitted article.

## Abbreviations

lncRNAs: Long noncoding RNAs
LUSC: Lung squamous cell carcinoma
LINC00174: Long intergenic nonprotein coding RNA 00174
miRNA: MicroRNA
RT-qPCR: Reverse transcription quantitative real-time polymerase chain reaction
NFIX: Nuclear factor IX
ceRNA: Competing endogenous RNA
NSCLC: Non-small-cell lung cancer
LUAD: Lung adenocarcinoma
ncRNAs: Noncoding RNAs
EMEM: Eagle's minimum essential medium
shRNAs: Short hairpin RNAs
NC: Negative control
cDNA: Complementary DNA
EdU: 5-Ethynyl-2′-deoxyuridine
TUNEL: Terminal-deoxynucleotidyl transferase mediated nick end labeling
FISH: Fluorescence in situ hybridization
WT: Wild-type
MUT: Mutated
RIP: RNA immunoprecipitation
SPF: Specific-pathogen free.

## Supplementary Materials

Supplementary Materials FISH assay probe sequence.

## References

[1] Siegel R. L., Miller K. D., Jemal A. (2017). Cancer statistics, 2017. *CA: a Cancer Journal for Clinicians*.

[2] Li S., Huang S., Peng S. B. (2005). Overexpression of G protein-coupled receptors in cancer cells: involvement in tumor progression. *International Journal f Oncology*.

[3] Antal C. E., Hudson A. M., Kang E. (2015). Cancer-associated protein kinase C mutations reveal kinase's role as tumor suppressor. *Cell*.

[4] Yang G., Lu X., Yuan L. (2014). LncRNA: a link between RNA and cancer. *Biochimica et Biophysica Acta*.

[5] Wang X., Zhang J., Wang Y. (2019). Long noncoding RNA GAS5-AS1 suppresses growth and metastasis of cervical cancer by increasing GAS5 stability. *American Journal of Translational Research*.

[6] Zhang Y., Hou Y. M., Gao F., Xiao J. W., Li C. C., Tang Y. (2019). lncRNA GAS5 regulates myocardial infarction by targeting the miR-525-5p/CALM2 axis. *Journal of Cellular Biochemistry*.

[7] Wu X., Xiao Y., Zhou Y., Zhou Z., Yan W. (2019). lncRNA SNHG20 promotes prostate cancer migration and invasion via targeting the miR-6516-5p/SCGB2A1 axis. *American Journal of Translational Research*.

[8] Zhang H. Y., Yang W., Zheng F. S., Wang Y. B., Lu J. B. (2017). Long non-coding RNA SNHG1 regulates zinc finger E-box binding homeobox 1 expression by interacting with TAp63 and promotes cell metastasis and invasion in lung squamous cell carcinoma. *Biomedicine & Pharmacotherapy = Biomedecine & Pharmacotherapie*.

[9] Sui J., Xu S. Y., Han J. (2017). Integrated analysis of competing endogenous RNA network revealing lncRNAs as potential prognostic biomarkers in human lung squamous cell carcinoma. *Oncotarget*.

[10] Tang R. X., Chen W. J., He R. Q. (2017). Identification of a RNA-Seq based prognostic signature with five lncRNAs for lung squamous cell carcinoma. *Oncotarget*.

[11] Shen Y., Gao X., Tan W., Xu T. (2018). STAT1-mediated upregulation of lncRNA LINC00174 functions a ceRNA for miR-1910-3p to facilitate colorectal carcinoma progression through regulation of TAZ. *Gene*.

[12] Zhi Q., Wan D., Ren R. (2021). Circular RNA profiling identifies circ102049 as a key regulator of colorectal liver metastasis. *Molecular Oncology*.

[13] Zhang X., Wang W., Zhu W. (2019). Mechanisms and functions of long non-coding RNAs at multiple regulatory levels. *International Journal of Molecular Sciences*.

[14] Zeng X. Y., Jiang X. Y., Yong J. H. (2019). lncRNA ABHD11-AS1, regulated by the EGFR pathway, contributes to the ovarian cancer tumorigenesis by epigenetically suppressing TIMP2. *Cancer Medicine*.

[15] Song Z., Zhang X., Lin Y., Wei Y., Liang S., Dong C. (2019). LINC01133 inhibits breast cancer invasion and metastasis by negatively regulating SOX4 expression through EZH2. *Journal of Cellular and Molecular Medicine*.

[16] Guo Z., He C., Yang F., Qin L., Lu X., Wu J. (2019). Long non-coding RNA-NEAT1, a sponge for miR-98-5p, promotes expression of oncogene HMGA2 in prostate cancer. *Bioscience Reports*.

[17] Xu Y., Li J., Wang P., Zhang Z., Wang X. (2019). LncRNA HULC promotes lung squamous cell carcinoma by regulating PTPRO via NF- *κ*B. *Journal of Cellular Biochemistry*.

[18] Shi J., Zhang Y., Qin B., Wang Y., Zhu X. (2019). Long non-coding RNA LINC00174 promotes glycolysis and tumor progression by regulating miR-152-3p/SLC2A1 axis in glioma. *Journal of Experimental & Clinical Cancer Research: CR.*.

[19] Zhao J. T., Chi B. J., Sun Y. (2020). LINC00174 is an oncogenic lncRNA of hepatocellular carcinoma and regulates miR-320/S100A10 axis. *Cell Biochemistry and Function*.

[20] Li B., Zhao H., Song J., Wang F., Chen M. (2020). LINC00174 down-regulation decreases chemoresistance to temozolomide in human glioma cells by regulating miR-138-5p/SOX9 axis. *Human Cell*.

[21] Niu Y., Tang G. (2019). miR-185-5p targets ROCK2 and inhibits cell migration and invasion of hepatocellular carcinoma. *Oncology Letters*.

[22] Yu H., Xu A., Wu B., Wang M., Chen Z. (2021). Long noncoding RNA NEAT1 promotes progression of glioma as a ceRNA by sponging miR-185-5p to stimulate DNMT1/mTOR signaling. *Journal of Cellular Physiology*.

[23] Ye L., Feng W., Weng H., Yuan C., Liu J., Wang Z. (2020). MAFG-AS1 aggravates the progression of pancreatic cancer by sponging miR-3196 to boost NFIX. *Cancer Cell International*.

[24] Xu Y. J., Zhou R., Zong J. F. (2019). Epstein-Barr virus-coded miR-BART13 promotes nasopharyngeal carcinoma cell growth and metastasis via targeting of the _NKIRAS2_ /NF-*κ*B pathway. *Cancer Letters*.

[25] Yang L., Yang Z., Yao R. (2018). miR-210 promotes progression of endometrial carcinoma by regulating the expression of NFIX. *International Journal of Clinical and Experimental Pathology*.

